RETRACTED

# Circulating miR-340-5p and miR-506-3p as Two Osteo-miRNAs for Predicting Osteoporosis in a Cohort of Postmenopausal Women

**DOI:** 10.1155/2023/7571696

**Published:** 2023-01-31

**Authors:** Zifeng Lu, Haiou Cao, Xiaoyin Hu

**Affiliations:** ^1^Department of Orthopedics (No. 1), Heilongjiang Beidahuang Group General Hospital, Harbin, Heilongjiang 150088, China; ^2^Department of Oncology (No. 6), Heilongjiang Beidahuang Group General Hospital, Harbin, Heilongjiang 150088, China; ^3^Department of Orthopedics, Shanghai LiQun Hospital, Shanghai, China

## Abstract

**Objective:**

An increasing risk of developing osteoporosis which is characterized by bone production weakness and microarchitectural deterioration is found among postmenopausal women. MicroRNAs (miRNAs) are secreted into the circulation from cells of various tissues in response to local disease severity including bone diseases. Herein, we set out to identify candidate miRNAs predictable for osteoporosis incidence in postmenopausal elderly women.

**Methods:**

The circulating miRNA expression profiles deposited in the dataset accessioned as GSE201543 were downloaded from the GEO database. The study included 176 postmenopausal women who underwent BMD testing, including 96 women reporting osteoporosis and 70 women reporting normal BMD. All subjects were submitted their serum samples for measurements of bone metabolism markers.

**Results:**

The miRNA expression profiles of the GSE201543 dataset were differentially analyzed and found 97 miRNAs being upregulated concomitantly with 31 miRNAs being downregulated in the serum samples between osteoporotic postmenopausal women and postmenopausal women with normal BMD. Osteoporotic postmenopausal women were demonstrated with elevated serum levels of miR-340-5p and miR-506-3p when compared to normal postmenopausal women. Pearson correlation analysis demonstrated that circulating miR-340-5p and miR-506-3p expressions were increased as BAP, *β*-CTx, and PINP levels increased, but osteocalcin and 25-(OH)VitD levels are declined in osteoporotic postmenopausal women. Results of the receiver operating characteristic (ROC) curve and the area under the ROC curve (AUC) showed circulating miR-340-5p and miR-506-3p expressions alone or combined together produced 0.843 AUC, 0.851 AUC, and 0.935 AUC, respectively, when used to predict the incidence of osteoporosis in postmenopausal women.

**Conclusion:**

Our work suggested that circulating miR-340-5p and miR-506-3p function as osteo-miRNAs in postmenopausal women and may serve as potential noninvasive biomarkers for the incidence of osteoporosis in postmenopausal women.

## 1. Introduction

Osteoporosis is a skeletal disease arising from a diseased condition that bone formation is overwhelmed by bone resorption and has a high morbidity rate among elderly individuals, particularly, women of postmenopausal age [1, 2]. Osteoporosis and subsequent fractures involve half of women and one-fifth of men who are aged more than 50 years worldwide, leading to substantial morbidity and an unsatisfactory quality of life [3]. Osteoporosis is characterized by bone production weakness along with microarchitectural deterioration leading to a higher risk of fracture [4]. The past half-century has witnessed the development of scanning modalities for BMD and bone microarchitecture measurements, such as dual-energy X-ray absorptiometry or quantitative CT [5]. The gradual imbalance between bone formation and resorption can be caused by multiple factors, including aging, estrogen deficiency, and prolonged immobilization, followed by disruption of normal apoptosis and autophagy with excessive inflammation [6]. Preventing the occurrence and minimizing the risk of fractures are the main goals of several pharmacological agents for osteoporosis management either by inducing bone formation or by reducing bone resorption, including zoledronic acid, calcitonin, and salmon calcitonin [7]. Interestingly, bone mineral density (BMD), osteoporosis, and osteoporotic fracture are shown to bind avidly to heritability [8]. However, it is still challenging to determine the genetic architecture, especially the genomic and molecular mechanisms contributing to osteoporosis.

RETRACTED

Detections of circulating microRNAs (miRNAs) as potential biomarkers for the risk of osteoporosis and subsequent fractures by next-generation sequencing (NGS) and global miRNA expression have recently attracted much attention [9]. miRNAs have the ability to post-transcriptionally regulate and silence target gene expression and thus play osteoclast differentiation and survival, as well as osteoblast-to-osteoclast communication [10]. For example, two miRNAs, miR-485-3p and miR-491-5p, were reported to protect osteoporotic postmenopausal women against vertebral fractures [11]. miR-340-5p is localized in 5q35 and has been demonstrated to target many genes, such as ROCK1, FHL2, and SKP2, and to regulate the relevant mechanisms involving several signaling pathways, such as JAK-STAT, and Wnt/*β*-catenin pathways, thus contributing to in the initiation of several diseases [12]. miR-506-3p was reported to regulate RAB3D expression and repress osteosarcoma cell proliferation and growth [13]. In the beginning, we analyzed the raw data sourced from the GSE201543 dataset and found that miR-340-5p and miR-506-3p were two osteoporosis-related miRNAs (osteo-miRNAs) among postmenopausal women. Herein, we set out to validate the diagnostic values of these two osteo-miRNAs as noninvasive biomarkers in osteoporotic postmenopausal women.

RETRACTED

## 2. Materials and Methods

### 2.1. Bioinformatics Analysis

The Gene Expression Omnibus (GEO, https://www.ncbi.nlm.nih.gov/gds) was thoroughly retrieved to acquire miRNA expression profiles associated with osteoporosis in postmenopausal women. The circulating miRNA expression profiles deposited in the dataset accessioned as GSE201543 were downloaded for further analysis. The GSE201543 dataset encompassed 10 serum samples being made up of 6 postmenopausal women with osteoporosis (sample labels: GSM6067330-GSM6067335) and 4 postmenopausal women without osteoporosis (sample labels: GSM6067336-GSM6067339) and generated on the GPL20712 platform (Agilent-070156 Human miRNA). Differentially expressed miRNAs in the serum sample between postmenopausal women with osteoporosis and postmenopausal women without osteoporosis must fulfill log2|fold change (FC)| > 2 and adjusted *p* < 0.05 by using the GEO2R bioinformatics tool [14]. The volcano maps and heatmaps were generated to present all differentially expressed miRNAs and expression diversity of representative differentially expressed miRNAs.

### 2.2. Study Subjects

The study included 176 postmenopausal women who underwent BMD testing at the Heilongjiang Beidahuang Group General Hospital between January 2021 and December 2022. The diagnosis of osteoporosis was confirmed based on the classification criteria of the World Health Organization (WHO) based on T-score of BMD testing [15]: T-scores not less than −1.0 were deemed as normal BMD, T-scores ranging from −1.0 to −2.5 as osteopenia, and T-scores not more than −2.5 as osteoporosis. Exclusion criteria for study subjects were as follows: complications such as rheumatoid arthritis or collagen, diabetes mellitus, endocrine disorders, and chronic liver diseases, which influence bone mass; systemic lupus erythematosus, metabolic and endocrine diseases, connective tissue disease, hyperthyroidism, spondylitis, bone tumors, or previous history of hormone replacement therapy, corticosteroid therapy, and stress hormones, which affect bone metabolism; previous history of bisphosphonates. Additionally, patients with common fractures, family history of bone disorder, or low physical activity, and mental illness were also excluded from the study. All included subjects were informed of the medical record review and study design and signed consent documents before data collection. The Ethics Committee of the Heilongjiang Beidahuang Group General Hospital approved and reviewed the study protocol.

RETRACTED

### 2.3. Human Serum Sample Collection

Blood samples (5 ml venous blood) were obtained from all subjects on the next day from 9:00 to 11:30 a.m. after an overnight fast to avoid potential diurnal influence. The serum was obtained following centrifugation (3000 r/min, 5 min) of blood samples and equally submitted for bone metabolism marker detection and RNA extraction, respectively.

### 2.4. BMD Measurements and Bone Metabolism Evaluation

BMD measurements of the femoral neck, lumbar spine, total hip, and 1/3 radius applied the DPX-MD dual-energy X-ray bone densitometry (LUNA, USA). The serum levels of bone alkaline phosphatase (BAP) and osteocalcin were measured with the aid of a colorimetric analyzer (Cobas Integra, Roche, Switzerland) using the immunoenzymetric assay kits (MicroVue BAP, USA) and immunoassay ELISA kits (MicroVue Osteocalcin, USA), respectively. The serum levels of *β*-carboxyl terminal peptide (*β*-CTx), propeptide of type I procollagen (PINP), and 25⁃hydroxyvitamin D (25-(OH)VitD) were detected using the patented electrochemiluminescence (ECLIA) method by a Cobas Integra colorimetric analyzer with the aid of kits (USCN Life Science, Wuhan, China).

### 2.5. RNA Extraction, cDNA Synthesis, and Quantitative Real-Time PCR (qRT-PCR)

Total RNA was extracted from the serum samples using TRIzol reagent (Invitrogen, USA). The reverse transcription was applied to the PrimeScript RT Master Mix (Takara, Japan). The PCR amplification of candidate miRNAs was carried out by the ABI 7300 machine (Applied Biosystems, USA) with the aid of the SYBR Green I Master Mix kit (Invitrogen, USA), with results presented by the 2^−ΔΔC^ method. The primer sequences for miR-340-5p, miR-506-3p, and the endogenous reference U6 are listed in Table 1.

### 2.6. Statistical Analysis

All data produced in the study were shown as mean ± standard deviation and submitted into the SPSS 21.0 software for statistical comparisons. The studied variables include age, BMI, menopause years, BMD of the femoral neck, lumbar spine, total hip, and 1/3 radius, and the serum levels of bone metabolism markers, circulating miR-340-5p and miR-506-3p expressions between osteoporotic women and normal postmenopausal women, were compared by using two independent sample *t*-test. Pearsom correlation analysis was applied to estimate associations between circulating miR-340-5p expression, miR-506-3p expression, and the studied independent variables in osteoporotic women. Osteoporosis diagnosis using miR-340-5p and miR-506-3p alone or in combination at a baseline expression level applied the receiver operating characteristic (ROC) curve and the area under the ROC curve (AUC). The level of *p* < 0.05 denoted a statistically significant difference.

RETRACTED

## 3. Results

### 3.1. The Demographics and Baseline Bone Parameters of Study Subjects

There were 176 postmenopausal women in this study, among which 96 postmenopausal women (54.55%) reported osteoporosis with *T*-score ≤ −2.5, 10 postmenopausal women (5.68) reported osteopenia with *T*-score ranging from −1.0 to −2.5, and 70 postmenopausal women (39.77%) reported normal *T*-score ≥ −1.0. Osteoporotic postmenopausal women exhibited decreased BMI, longer years of menopause, declined BMD in the femoral neck, lumbar spine, total hip, and 1/3 radius, lower *T*-scores of the femoral neck and lumbar spine compared with normal postmenopausal women (*p* < 0.001, Table 2). With regard to baseline bone parameters, it was found that the serum levels of BAP, *β*-CTx, and PINP were higher, but the serum levels of osteocalcin, 25-(OH)VitD, were lower in osteoporotic postmenopausal women than normal postmenopausal women (*p* < 0.001, Figure 1).

### 3.2. High Circulating miR-340-5p and miR-506-3p in Osteoporotic Postmenopausal Women

To study molecular alternations related to the incidence of osteoporosis in postmenopausal women, we submitted miRNA expression profiles of the GSE201543 dataset for differential analysis and found 97 miRNAs being upregulated concomitantly with 31 miRNAs being downregulated in the serum samples between osteoporotic postmenopausal women and postmenopausal women with normal BMD. The top 5 upregulated circulating miRNAs ranked by *p* values in osteoporotic postmenopausal women were miR-4527, miR-5186, miR-340-5p, miR-506-3p, and miR-4770 (Table 3). After reviewing relevant literature about these miRNAs in osteoporosis, we selected miR-340-5p and miR-506-3p for further detection in the serum samples of 96 osteoporotic postmenopausal women and 70 normal postmenopausal women. Osteoporotic postmenopausal women were demonstrated with upregulated miR-340-5p and miR-506-3p when compared to normal postmenopausal women (*p* < 0.001, Figure 2).

### 3.3. Circulating miR-340-5p and miR-506-3p Correlated with Bone Metabolism Markers in Osteoporotic Postmenopausal Women

Pearson correlation analysis demonstrated that circulating miR-340-5p and miR-506-3p expressions were increased as BAP, *β*-CTx, and PINP levels increased, but osteocalcin and 25-(OH)VitD levels declined in osteoporotic postmenopausal women (*p* < 0.001, Figure 3 and Table 4).

### 3.4. The Diagnostic Values of Circulating miR-340-5p and miR-506-3p in Osteoporotic Postmenopausal Women

The diagnostic performance for circulating levels of miR-340-5p and miR-506-3p in clinical serum samples for osteoporotic postmenopausal women was determined using the AUC. Results showed that circulating miR-340-5p and miR-506-3p expressions produced 0.843 AUC (Figures 4(a) and 4(b), *p* < 0.01) and 0.851 AUC (*p* < 0.01), respectively. Additionally, we found a much stronger diagnostic value for the incidence of osteoporosis in postmenopausal women with an AUC of 0.935 (*p* < 0.001, Figure 4(c)) produced by circulating miR-340-5p and miR-506-3p levels in combination compared to a single miRNA (*p* < 0.01). Circulating miR-340-5p expression conferred 72.90% sensitivity and 87.10% specificity for osteoporotic postmenopausal women. Circulating miR-506-3p expression conferred 74.00% sensitivity and 85.70% specificity for osteoporotic postmenopausal women. Circulating miR-340-5p and miR-506-3p combined together conferred 84.40% sensitivity and 92.90% specificity for osteoporotic postmenopausal women.

RETRACTED

## 4. Discussion

Osteoporosis represents a common public health burden among elderly individuals, especially among postmenopausal women. Considering excellent stability, tissue specificity, as well as easy detection of circulating miRNAs, they have been widely applied for the prediction and early diagnosis of human diseases, including metabolic bone disease [16]. miRNAs are shown to be closely associated with osteoblast and osteoclast differentiation and survival in the context of bone formation [17]. We performed differential expression analysis using miRNA expression profiles of the GSE201543 dataset and found the top 5 upregulated circulating miRNAs ranked by *p* values in osteoporotic postmenopausal women compared with postmenopausal women with normal BMD, miR-4527, miR-5186, miR-340-5p, miR-506-3p, and miR-4770. Clinical validation demonstrated acceptable diagnostic values of miR-340-5p and miR-506-3p alone or in combination for osteoporosis incidence among postmenopausal women.

Bone turnover markers can be employed alone or in combination with other bone parameters to evaluate bone resorption and bone formation in aged postmenopausal women [18]. As demonstrated by Thejaswi et al., the BAP level was helpful as a screening biomarker to predict osteoporosis in postmenopausal women [19]. *β*-CTx as a key resorption marker was shown to be more predictive for fracture risk than formation markers in very elderly women [20]. Serum PINP is designated as an important bone formation marker in osteoporosis, and it, with CTX, was commonly utilized to evaluate the offset of drug action after bisphosphonate therapy [21]. Osteocalcin is considered as a bone matrix protein, and osteoporosis patients exhibited a decreased osteocalcin level when compared to those with normal BMD [22]. A decreasing level of serum 25-(OH)VitD is regarded as one of the most events predicting the incidence of fractures in elderly women [23]. In the study, the levels of BAP, *β*-CTx, and PINP notably elevated, and the levels of osteocalcin and 25-(OH)VitD significantly declined in osteoporotic postmenopausal women compared with normal postmenopausal women.

RETRACTED

It is believed that molecular alternations were associated with bone metabolism. We found that osteoporotic postmenopausal women were demonstrated with elevated serum levels of miR-340-5p and miR-506-3p when compared to normal postmenopausal women, and circulating levels of miR-340-5p and miR-506-3p had positive correlations with the serum levels of BAP, *β*-CTx, and PINP, but negative correlations with the serum levels of osteocalcin and 25-(OH)VitD in osteoporotic postmenopausal women. A study of type I diabetes found high expression of miR-340-5p proportional to inflammatory cytokine-stimulated *β* cell damage [24]. The study reported by Du et al. showed that miR-340-5p inhibition could increase *β*-catenin expression and thus promote osteogenesis of bone marrow-derived mesenchymal stem cells [25]. Loss of miR-340-5p was also shown to enhance the levels of ALP, osteocalcin, collagen-I, and RUNX2 and increase calcium deposition, thus promoting osteogenesis of MC3T3-E1 [26]. miR-506-3p could inhibit osteogenic differentiation by modulating bone morphogenetic protein 7 [27]. All these previous reports showed similar results as our study, and thus, we believed that high circulating 340-5p and miR-506-3p expression may be linked with the incidence of osteoporosis among postmenopausal women.

In conclusion, the study supports the notion that circulating miR-340-5p and miR-506-3p along with bone turnover markers such as BAP, *β*-CTx, PINP, osteocalcin, and 25-(OH)VitD as potential diagnostic biomarkers for the occurrence of osteoporosis in postmenopausal women. However, further investigations with RNA sequencing or miRNA arraying will be performed to identify more specific miRNAs as diagnostic biomarkers for postmenopausal osteoporosis. Further investigations will also focus on miRNA control of mRNA in bone metabolism regulation of miR-340-5p and miR-506-3p, as well as more functional studies using ovariectomized mice.

## Figures and Tables

**Figure 1:** The serum levels of baseline bone parameters between osteoporotic postmenopausal women (*n* = 96) and postmenopausal women with normal BMD (*n* = 70). ^*∗*^*p* < 0.05, compared with postmenopausal women with normal BMD (by the unpaired *t*-test).

**Figure 2:** Circulating miR-340-5p and miR-506-3p expressions in clinical samples between osteoporotic postmenopausal women (*n* = 96) and postmenopausal women with normal BMD (*n* = 70). ^*∗*^*p* < 0.05, compared with postmenopausal women with normal BMD (by the unpaired *t*-test).

RETRACTED

**Figure 3:** Correlation analysis between circulating miR-340-5p, miR-506-3p, and bone metabolism markers in osteoporotic postmenopausal women (*n* = 96).

**Figure 4:** The diagnostic values of circulating miR-340-5p (a) and miR-506-3p (b) alone or combined together (c) in osteoporotic postmenopausal women (*n* = 96).

**Table 1:** The primer sequences for miR-340-5p, miR-506-3p, and the endogenous reference U6 used for qRT-PCR.

Name	Primer sequences (5′-3′)
miR-340-5p	Forward: 5′-CTGGTAGGTTATAAAGCAATGA-3′
	Reverse: 5′-TCAACTGGTGTCGTGGAG-3′

miR-506-3p	Forward: 5′-TAAGGCACCCTTCTGAGTAGA-3′
	Reverse: 5′-GCGAGCACAGAATTAATACGAC-3′

U6	Forward: 5′-GTGCTCGCTTCGGCAGCACAT-3′
	Reverse: 5′-TACCTTGCGAAGTGCTTAAAC-3′

**Table 2:** The demographics and baseline bone parameters of study subjects.

Name	Osteoporosis (*n* = 96)	Normal (*n* = 70)	*p* value
Age (year)	64.88 ± 4.30	63.81 ± 3.63	0.093
BMI (kg/m^2^)	22.65 ± 2.58	24.75 ± 3.70	<0.001
Menopause year	9.92 ± 3.30	8.68 ± 2.40	0.008
BMD femoral neck (g/cm^2^)	0.62 ± 0.29	0.76 ± 0.41	0.018
*T*-score for femoral neck	−2.63 ± 0.68	0.34 ± 0.43	<0.001
BMD lumbar spine (g/cm^2^)	0.69 ± 0.47	0.98 ± 0.70	0.003
*T*-score for lumbar spine	−2.81 ± 0.95	0.71 ± 1.22	<0.001
BMD total hip (g/cm^2^)	0.71 ± 0.46	0.86 ± 0.73	0.043
BMD 1/3 radius (g/cm^2^)	0.50 ± 0.35	0.69 ± 0.20	<0.001

BMI, body mass index; BMD, bone mineral density.

**Table 3:** The top 5 upregulated circulating miRNAs ranked by *p* values in osteoporotic postmenopausal women after analyzing miRNA expression profiles of the GSE201543 dataset.

ID	Log2FC	*p* value
hsa-miR-4527	6.42075	1.03*E* − 09
hsa-miR-5186	6.568372	1.29*E* − 09
hsa-miR-340-5p	5.796601	1.57*E* − 09
hsa-miR-506-3p	5.707624	1.57*E* − 09
hsa-miR-4770	5.797031	1.68*E* − 09

FC, fold change.

**Table 4:** Pearson correlation analysis of circulating miR-340-5p, miR-506-3p, and bone metabolism markers in osteoporotic postmenopausal women.

Bone metabolism markers	Circulating miRNA	
	miR-340-5p	miR-506-3p
BAP	*r* (95% CI) = 0.635 (0.498–0.741)	*r* (95% CI) = 0.552 (0.395–0.677)
*β*-CTx	*r* (95% CI) = 0.445 (0.269–0.593)	*r* (95% CI) = 0.405 (0.223–0.560)
PINP	*r* (95% CI) = 0.489 (0.320–0.628)	*r* (95% CI) = 0.352 (0.163–0.516)
Osteocalcin	*r* (95% CI) = −0.715 (−0.801–0.601)	*r* (95% CI) = −0.417 (−0.570–0.236)
25-(OH)VitD	*r* (95% CI) = −0.436 (−0.585–0.258)	*r* (95% CI) = −0.378 (−0.538–0.192)

BAP, bone alkaline phosphatase; *β*-CTx, *β*-carboxyl terminal peptide; PINP, propeptide of type I procollagen; 25-(OH)VitD, 25⁃hydroxyvitamin D.

RETRACTED

## Data Availability

The GSE201543 dataset was downloaded from the Gene Expression Omnibus database (GEO, https://www.ncbi.nlm.nih.gov/geo) that is a public database. Other data supporting this study are included within the article.
